The article "Logistics Distribution Path Optimization Algorithm Based on Intelligent Management System" was retracted in 2023. Reasons: unreliable results or conclusions; concerns about the data; concerns about the peer review; concerns about the citations.

# Logistics Distribution Path Optimization Algorithm Based on Intelligent Management System

**DOI:** 10.1155/2022/3699990

**Published:** 2022-09-26

**Authors:** Foshang Li

**Affiliations:** School of Business, Jilin Business and Technology College, Changchun 130507, Jilin, China

## Abstract

There are three key points in logistics distribution: the distribution vehicle, the amount of goods, and the distribution path. Comprehensive calculation and optimization of these three parameters can plan a reasonable and efficient distribution scheme, especially the distribution path. This study aims to study the method of optimizing the logistics distribution path and strives to find the optimal distribution scheme and the shortest path, which can reduce the distribution error rate, distribution time, and labor costs, thus realizing intelligent management. In this study, intelligent management methods such as radio-frequency identification technology and ant colony algorithm are proposed to optimize the logistics distribution path and realize the safe and efficient logistics distribution. The experimental results of this study show that for the current logistics distribution, the RFID system has a positioning rate of close to 100% when the number of fixed points reaches about 300, and almost all accurate positioning is achieved. The ant colony algorithm can also accurately find the shortest distance after selecting appropriate parameters, which is about 200 meters away from the actual shortest distance.

## 1. Introduction

With the continuous improvement of the scope and form of e-commerce, logistics has become more and more important, which has become one of the important points of competition in various industries of e-commerce. With the maturity of the logistics market, the requirements for the quality and punctuality of logistics services are getting higher and higher, and logistics distribution is the key to improving the quality and punctuality of logistics services. Optimizing distribution paths to realize intelligent management not only reduces capital investment and improves distribution efficiency but also realizes logistics information sharing, which can maintain close data exchange with customers and improve customers' sense of use.

Intelligent management is a software service IT platform developed based on the Internet, which can realize resource virtualization and parallel computing. It can also intelligently process massive data, with low latency, high availability, and easy expansion, effectively improving resource utilization. It reduces costs, and the computing power far exceeds the capabilities of typical virtualization solutions, so intelligent management can augment the logistics and distribution methods currently on the market. It can optimize logistics distribution routes by meeting the requirements of new distribution forms such as joint distribution across multiple distribution centers. Based on the above analysis, this study introduces an intelligent management system. A logistics distribution path optimization model is established, which can support the optimization of logistics distribution network, so as to realize the real-time sharing of logistics information, resources, and functions, so that enterprises can reduce logistics costs and make scientific management decisions. By introducing an intelligent management system to optimize the logistics distribution path and establish an optimization model, the real-time sharing of logistics information and resources between customers and merchants is realized. Enterprises can also reduce logistics input costs and make scientific management decisions.

This study proposes two methods: RFID technology and ant colony algorithm. Through experiments to measure the accuracy of fixed points and find the shortest path, it is concluded that the method in this study can accurately locate items on the logistics distribution path, shorten the distribution time, and reduce the input cost. The innovation of this study is as follows: radio-frequency identification technology uses wireless signals for noncontact information transmission, real-time sharing of logistics information (including items in motion), and accurate logistics positioning. Ant colony algorithm bionic ants are used to find the shortest path in logistics distribution and the shortest distance between two selected locations and maximize the shortening of logistics time.

## 2. Related Work

At present, with the booming development of commerce, people's life and work are gradually dependent on the logistics industry. In order to improve the logistics distribution, scholars have carried out research on the logistics industry. Among them, Yang studied the common distribution methods of urban logistics in the e-commerce environment and considered the dynamic uncertainty of the urban road network on the basis of the optimization of the distribution path [1]. Wu studied how to enable vehicles to upload their status to a cloud-based traffic control center (TCC) in real time and how to perform global optimized path planning and return the planning results to the requester to improve traffic congestion [2]. Sun studied the route optimization and improved genetic algorithm of aviation logistics distribution center [3]. Xiaoyan analyzed the path method of agricultural product logistics and distribution B2C mode under the e-commerce mode [4]. Speranza reviews the history of issues in transportation and logistics and the contribution of OR and technological developments and discusses future trends in the field and potential OR contributions [5]. It is not difficult to find that there are many application fields after the optimization of the logistics distribution path, and the optimization technology can also be extended to other industries, but these studies do not introduce much about the intelligent management system.

Researches on intelligent management systems are as follows: George studied the problem of setting pedestrian signals at roundabouts to improve the traffic system through artificial intelligence [6]. Hamidi studied the role of intelligent traffic management in emergency-related transportation including psychological [7]. Karimanzira studied the application of intelligent management systems in integrating digital technologies in aquaculture production and processing systems to increase consumer trust in aquaculture products [8]. Zheng studied the architecture and several technical issues of the intelligent management system and came to the conclusion that the adaptive behavior of the system shows that the system is superior to the mainstream system [9]. Wang studied the digital twin and cloud collaboration problem of intelligent battery management system [10]. Through the research on these two aspects, the understanding of intelligent management system and logistics distribution path will be deepened, but these studies are not highly relevant to the application of intelligent management in logistics management. The article strives to use intelligent management to optimize all aspects of the delivery process of goods, so as to improve the efficiency of delivery and the safety of goods.

## 3. Logistics Distribution Route Optimization Scheme Based on the Intelligent Management System

### 3.1. Optimization Method of Logistics Distribution Path

With the rapid development of B2B e-commerce, the development of logistics and distribution has also become a top priority, but at present, logistics and distribution are facing many problems. For example, logistics information can only be displayed at a fixed point and the infrastructure is relatively backward. The professional talents to improve the development of the logistics industry are relatively lacking. The input cost and delivery time need to be strengthened. The delivery speed and completion efficiency of the delivery system affect delivery costs and customer satisfaction. Meanwhile, the traditional distribution system is not sensitive to emergency intervention, which often causes some losses and reduces the reputation of logistics.

Aiming at these problems, the optimization methods designed in this study are as follows: an intelligent logistics warehouse management system based on RFID technology can help merchants to efficiently manage logistics warehouses online. It is a complete system that integrates functions such as collection and delivery management, warehouse management, cargo transportation and distribution, and cargo tracking, realizing the informatization and intelligence of the system. It can help logistics enterprise managers make real-time and scientific decisions, reduce logistics costs, and improve logistics distribution efficiency for logistics enterprises [11]. Its system frame diagram is shown in Figure 1.

In addition, the ant colony algorithm aims to find the shortest path for logistics distribution. After many cycles in the experiment, the flowchart of realizing the shortest path selection is shown in Figure 2.

This study designs and uses radio-frequency identification technology and ant colony algorithm to solve the problems in the current logistics distribution, improve the efficiency of logistics distribution, reduce time and cost consumption, and promote the development of the logistics industry.

### 3.2. Fixed-Point Precise Positioning Realized by RFID Technology

Radio-frequency identification technology is a noncontact automatic identification technology, which uses radio-frequency signals to realize noncontact information transmission through spatial coupling and achieves the purpose of identification through the transmitted information, and the identification work requires manual intervention.

RFID technology is widely used in product identification, tracking, positioning, and warehousing in the field of logistics. An RFID system usually consists of a reader, an electronic tag, an antenna, and a computer-controlled terminal. The working principle of RFID is shown in Figure 3.

RFID has strong positioning and identification capabilities, which can penetrate special features that cannot be identified by barcodes, such as ice, snow, fog, and dust. Meanwhile, the identification speed of RFID is also very fast, and the electronic tag can be reused and can take on a variety of shapes. Considering the above advantages, RFID is widely used in object recognition and short-range positioning applications. Because RFID technology also has certain shortcomings, the fusion of WSN and RFID technology is used for target positioning. This not only fully demonstrates the characteristics of wireless multihop communication and the configuration of the network itself but also achieves target localization with efficient identification, low energy consumption, and low system cost [12].

WSID system structure integrates hardware architecture, protocol stack, network architecture, network management, and operating system, which has the advantages of wireless sensor network and RFID technology. The multidirectional and organically integrated WSID network not only has the noncontact rapid identification and positioning capabilities of RFID but also has the large-scale deployment of WSN, dynamic topology, self-configured routing, application-specific functions, environmental awareness, and monitoring capabilities [13]. Therefore, WSID network positioning technology has great potential in the field of logistics. The structure of the WSID network positioning system is shown in Figure 4.

The figure is composed of people, vehicles, couriers, WSID nodes, WSID relay nodes, WSID gateways, WSID base stations, and local terminals, and the process is simple and clear. Many deployments in the positioning system block diagram are WSID nodes for communication using a wireless multihop approach. Nodes can be used on any monitoring target. Position accuracy can also be expressed as the position error of the difference between the measured position and the actual position of the target node. Position error is divided into absolute error and relative error. The absolute error refers to the mean square error between the measured coordinate value and the actual coordinate value of the target node. The mean square error value between the relative errors represents the ratio of the absolute error to the communication radius of the beacon node [14]. The absolute error expression is as follows:

(1) $$\begin{array}{c} error=\overset{n}{\underset{i=1}{\sum }}\left|\sqrt{{\left(a_{i}-{\bar{a}}_{i}\right)}^{2}+{\left(b_{i}-{\bar{b}}_{i}\right)}^{2}}\right|/n\text{.} \end{array}$$

In formula (1), the actual and measured positions of target node *i* are denoted by $\left(\bar{a_{i}},\bar{b_{i}}\right)$ and (*a*_*i*_, *b*_*i*_), respectively. The relative error expression is as follows:

(2) $$\begin{array}{c} {error}^{\prime }=\overset{n}{\underset{i=1}{\sum }}\left|\sqrt{{\left(a_{i}-{\bar{a}}_{i}\right)}^{2}+{\left(b_{i}-{\bar{b}}_{i}\right)}^{2}}\right|/nr\times 100\%\text{.} \end{array}$$

The communication radius of the beacon node is represented by *r* in the formula. The positioning accuracy is the main performance index used to evaluate the positioning algorithm. The smaller the positioning error is, the higher the positioning accuracy will be.

According to different positioning methods, positioning algorithms can be divided into many kinds. The core problem of the distance measurement algorithm is that the beacon node measures the distance information between itself and the target node and directly converts the distance information into the target node information [15]. The core problem of the distance positioning algorithm is the accurate measurement of the distance between nodes. The method of measuring the accurate distance information between nodes is the most important problem of the positioning algorithm based on distance measurement. Ranging technology includes four commonly used technologies: RSSI, TOA, TDOA, and AOA. The RSSI ranging technology converts the signal strength received by the node into the distance in a specific model. The accuracy of the distance usually depends on the accuracy of the model and the stability of the RF signal [16]. The signal is attenuated during propagation. In real-world applications, distance is usually measured using a simplified gradient model, which is expressed as follows:

(3) $$\begin{array}{c} P_{R}\left(c\right)=P_{L}\left(c_{0}\right)-10\eta lg\left(c/c_{0}\right). \end{array}$$

In formula (3), *P*_*R*_(*c*) indicates the received signal strength from signal transmitter *c*, and *P*_*L*_(*c*_0_) indicates the received signal strength from signal transmitter *c*_0_. *c*_0_ indicates the reference distance between the signal receiver and the transmitter. The road strength loss index is represented by *η*, which represents the energy loss value during the transmission process. The more twists and turns in the process and the more obstacles are, the greater the value of *η* will be. Therefore, when the distance gradually increases, the signal transmission power will gradually decrease. Formula (3) can be simplified as follows:

(4) $$\begin{array}{c} P_{R}\left(c\right)=D-10\eta lg\left(c\right). \end{array}$$

It can be written in RSSI form as follows:

(5) $$\begin{array}{c} RSSI=D-10\eta lg\left(c\right). \end{array}$$

Formula (5) expresses the relationship that exists between the received signal strength and the signal propagation distance. In general, as long as the characteristics of the radio-frequency equipment and the signal acceptance strength are known, the distance between the transmitter and the receiver can be calculated [17].

The TOA technology is used to calculate the propagation distance of electromagnetic waves from the transmitter to the receiver. Assuming that the propagation time of the electromagnetic wave from the transmitter to the receiver is *t*, the propagation distance is expressed as follows:

(6) $$\begin{array}{c} d=t*c. \end{array}$$

In formula (6), *d* represents the propagation distance of the electromagnetic wave, *t* represents the propagation time, and *c* represents the propagation speed of the electromagnetic wave, in which the numerical size is 3 × 10^8^m/s. Since the propagation speed of electromagnetic waves is as fast as the speed of light, the accuracy of this method of measuring distance mainly depends on the accuracy of the calculation time. If it is not careful, the error will be very large [18].

Supposing that *n* readheads, *t* georeferenced tags, and *q* moving object tags are located in the environment, the reader is always in continuous working mode. Among them, P is defined as the energy value set of positioning tags received by the reader and *Q* is defined as the energy value set of reference tags received by the reader. The expressions are as follows:

(7) $$\begin{array}{c} P=\left(P_{1},P_{2},P_{3},{...P}_{n}\right), \end{array}$$

(8) $$\begin{array}{c} Q=\left(Q_{1},Q_{2},Q_{3},{...Q}_{n}\right). \end{array}$$

The Euclidean distance of each positioning label to the reference label can be expressed as follows:

(9) $$\begin{array}{c} E_{j}=\sqrt{\overset{n}{\underset{i=1}{\sum }}{\left(Q_{i}-P_{i}\right)}^{2}},i\in \left(1,2,3,...n\right),j\in \left(1,2,3,...m\right). \end{array}$$

Formula (9) expresses the relative strength of the placement label and the reference label. Each set of targeting tags has a set of matching relative intensity values, which is expressed as follows:

(10) $$\begin{array}{c} E=\left(E_{1},E_{2},E_{3},...E_{m}\right). \end{array}$$

Then, the *t* minimum values are obtained from *E*, and the K nearest neighbor method is used to estimate the coordinates of the identified position, whose expression is as follows:

(11) $$\begin{array}{c} \left(a,b\right)=\overset{t}{\underset{i=1}{\sum }}\omega_{i}\left(a_{i},b_{i}\right)\text{.} \end{array}$$

In formula (11), *ω*_*i*_ represents the weight. According to experience, the following formula can be obtained:

(12) $$\begin{array}{c} \omega_{i}=\frac{1/E_{m}^{2}}{\overset{t}{\underset{i=1}{\sum }}1/E_{m}^{2}}. \end{array}$$

Formula (12) reflects the main influencing factors including proximity weight, location, and the number of reference labels.

Radio-frequency identification (RFID) technology is a high-tech technology that can collect and process information in real time, quickly and accurately when applied. In order to realize the automatic identification of stationary and moving objects in logistics distribution, it mainly depends on the principle of the technology's radio-frequency signal and its spatial coupling and transmission characteristics. It is the first step in realizing information standardization. The principle is to use the radio-frequency signal and its spatial coupling and transmission characteristics to realize the automatic identification of stationary and moving objects. This technology is used in logistics and distribution, which can make the goods automatically identify the destination of the goods at each station from receipt to delivery. This greatly saves the time for sorting goods, labor costs, and time costs. Moreover, for some fragile or special commodities, alternative management can be identified to avoid damage to the items, which not only improves the efficiency of goods distribution but also ensures the safety of people's items.

### 3.3. Optimal Path of Logistics Distribution Based on Ant Colony Algorithm

Ant colony algorithm is a biological optimization probabilistic algorithm. Based on the evolution process of information exchange between ant colonies, the optimal solution is finally found. It is divided into the adaptation stage and cooperation stage. It is named after the ant's search for the shortest path in life. In reality, the ability of an ant may be very small. There may be obstacles to finding the shortest path, but the ant colony has a high degree of self-organization and will divide and cooperate with each other. If the entire ant colony is combined with the pheromone of each ant in the colony, it can cooperate to complete complex behaviors and exchange the path information they have traveled with each other, finding a shortest path [19]. Its image simulation diagram is shown in Figure 5.

As shown in the figure, there are two routes from the ant colony to bypass the obstacle to reach the food, namely, BA and CA, and the path lengths are 5 and 7, respectively. Ants convey certain information by leaving pheromones as markers on the path they traveled. When passing a certain number of times, most ants choose the shorter path on the left.

In the mathematical model of the ant colony algorithm, assuming that *ε*_*ij*_(*t*) represents the concentration of pheromones left by the ants at path (*i*, *j*) at time *t*, and *s*_*i*_(*t*) represents the number of ants located at a place *i* at time *t*, the formula for calculating the total number of ants is as follows:

(13) $$\begin{array}{c} z=\overset{n}{\underset{i=1}{\sum }}s_{i}\left(t\right). \end{array}$$

In the above formula, *n* represents the place with the number of ants, which is classified as a TSP model. In the beginning, the pheromone concentration of each road is the same, which is a constant value.

(14) $$\begin{array}{c} P_{ij}^{a}\left(t\right)=\left\{\begin{array}{c} \frac{{\left[\varepsilon_{ij}\left(t\right)\right]}^{\alpha }\cdot {\left[\eta_{ia}\left(t\right)\right]}^{\beta }}{\sum_{s\in {alloesd}_{a}}{\left[\varepsilon_{is}\left(t\right)\right]}^{\alpha ∙}\cdot {\left[\eta_{is}\left(t\right)\right]}^{\beta }\;}\;,j\in {alloesd}_{a},\\ 0,otherwise. \end{array}\right. \end{array}$$

In the above formula, *P*_*ij*_^*a*^(*t*) represents the state transition probability of ant a from location *i* to location *j*, *ε*_*is*_(*t*) represents the pheromone concentration left by the ants at the path at time *t*, and *α* represents the information heuristic factor, which is used to indicate the relative importance of the trajectory and reflect the role of the information accumulated by the ants during the migration process. *β* represents the expected heuristic factor, which is used to indicate the visibility and the degree of heuristic information that reflects the ant's assessment of movement when choosing a route. According to the greedy law, the higher the value is, the closer the probability of state transition is [20]. *η*_*ij*_(*t*) refers to the heuristic information value, and its TSP model expression is as follows:

(15) $$\begin{array}{c} \eta_{ij}\left(t\right)=\frac{1}{d_{ij}}. \end{array}$$

In the above formula, *d*_*ij*_ represents the distance between two adjacent places *i* and *j*, and the smaller the distance, the greater the heuristic information value. For ant a, the probability of arriving at destination city *j* is higher. Since there are many pheromones left by ants in each path process, in order to avoid residual elements that may hide useful information in the information, it needs to be updated after the ant colony process [21]. Pheromone can be adjusted according to the following formula:

(16) $$\begin{array}{c} \varepsilon_{ij}\left(t+n\right)=\left(1-\rho \right)\cdot \varepsilon_{ij}\left(t\right)+∆\varepsilon_{ij}\left(t\right),\\ ∆\varepsilon_{ij}\left(t\right)=\overset{m}{\underset{a=1}{\sum }}∆\varepsilon_{ij}^{a}\left(t\right). \end{array}$$

In the formula, the pheromone volatility coefficient is represented by *ρ*, and the residual information factor is represented by 1 − *ρ*. The information increment of all information in a circular path is represented by ∆*ε*_*ij*_(*t*), and the increment of the pheromone left by the ath ant in the path is represented by ∆*ε*_*ij*_^*a*^(*t*).

At present, in order to improve the solution speed of the ant colony algorithm, through the research on the ant colony path, the ant colony algorithm is proposed as an optimal solution to make it more attractive for the next iteration search. For each iteration of ants, additional pheromone concentrations are added to the optimal solution path so far, and when an ant finds the current optimal solution, such an ant is called an elite ant. Each time the ant repeats, adding an additional concentration of pheromone to the best solution so far, the ant that finds the optimal path is called an elite ant [22]. Assuming that the optimal path is 1 and its length is *L*, its expression is as follows:

(17) $$\begin{array}{c} \varepsilon_{ij}\left(t+n\right)=\left(1-\rho \right)*\varepsilon_{ij}\left(t\right)+\overset{m}{\underset{a=1}{\sum }}∆\varepsilon_{ij}^{a}+∆\varepsilon_{ij},\\ {∆\varepsilon }_{ij}=\left\{\begin{array}{c} \frac{\sigma }{L},\\ 0. \end{array}\right. \end{array}$$

Among them, *σ* is a setting parameter, which is mainly used to define the size of the weight. Experimental results show that good choices can help ants find better solutions and reduce convergence time. However, if the value of *σ* is too large, making the addition of the current optimal solution too large, the ant will choose this path. While the probability of choosing another path would be very low, the ants would converge quickly, repeating the same path as quickly as possible and moving on without finding a better practical solution.

The elite ant system also has a disadvantage. When finding the optimal path in an infinite loop, the ants tend to choose the optimal path. Therefore, the concentration of pheromone on other paths is not high, so that most ants only concentrate on the local optimal path and cannot quickly find the global optimal path [23]. Aiming at this problem, the improved regular expression is as follows:

(18) $$\begin{array}{c} \varepsilon_{ij}\left(t+n\right)=\rho *\varepsilon_{ij}\left(t\right)+\overset{\sigma -1}{\underset{a=1}{\sum }}∆\varepsilon_{ij}^{a}+∆\varepsilon_{ij},\\ ∆\varepsilon_{ij}^{a}=\left\{\begin{array}{c} \left(\sigma -a\right)\frac{1}{L^{a}},\\ 0, \end{array}\right.\\ ∆\varepsilon_{ij}=\left\{\begin{array}{c} \frac{\sigma }{L},\\ 0. \end{array}\right. \end{array}$$

In the formula, the ant sorting number is represented as a, and the accumulated value of the pheromone released by the ath ant on the path it passes through is represented as ∆*ε*_*ij*_^*a*^. By selecting the appropriate value, by adding the advantages and disadvantages of information elements on the basis of the existing optimal solution, the possibility of ants choosing the optimal solution is increased, and the optimal solution can be effectively utilized.

## 4. Experiment on Optimizing Logistics Distribution Path Based on Intelligent Management Systems

### 4.1. Experiment Results of RFID Technology

Using radio-frequency identification technology, when the target node enters the monitoring area, if the beacon node is constantly active, the target node will be continuously monitored, and the ranging information of the target node will be transmitted to the sink node. In this experiment, according to the different time intervals used, the positioning errors of all the test algorithms are collected, as shown in Figure 6.

As can be seen from the above figure, the use of radio-frequency identification technology in logistics management to identify the specific location error rate of the goods is very low, which means that the accuracy is very high, and the error is controlled to below 10%. The two lines of the measured distance and the real distance result graph almost overlap, indicating that the distance difference is almost the same. It can be seen that the position of each item can be accurately located when picking up the goods, thereby reducing the search time. In this way, less time can be consumed in a day, the efficiency of incoming and outgoing shipments can be improved, and logistics information can be shared with customers in real time. The customer knows the specific point of the goods, which also improves the safety of the goods.

For different numbers of beacon nodes, the positioning rate and the connectivity of the message network will also be different during identification. The specific experimental data during the experiment is shown in Figure 7.

With the increase of the number of beacon nodes, the location rate of the test also increases, the location accuracy is higher, and the connectivity between nodes is also higher. Among the factors affecting the positioning algorithm, in addition to the number of beacon nodes, there is also the communication distance of beacon nodes. In this experiment, the communication distance is kept different, other experimental environments are the same, and the KF algorithm, the APIT algorithm, and the SGM algorithm are used for testing. The experimental results are shown in Figure 8.

The above figure describes the change of the positioning error of the three algorithms when the communication distance of the beacon node is from 40 meters to 100 meters. It can be seen that the smaller the distance, the greater the positioning error rate. Combined with the experiment, it can be found that the radio-frequency identification technology can effectively identify the fixed point position within a short distance. The greater the quantity of logistics goods and the greater the communication distance within a certain range, the higher the positioning accuracy. The application of this technology in logistics stations is very suitable, especially during online shopping festivals such as Double Eleven and 618, the more obvious the advantages are. When the logistics pressure is too great, the manpower cannot work, and it is the place where technology comes into play.

### 4.2. Experimental Results of Ant Colony Algorithm

The ant colony algorithm is inspired by the actual behavior of the ant colony in reality. Ant individuals are small and their behavioral abilities are also weak, but when ants are combined, they can form a highly structured group, which enables a group of ants to work together to complete a difficult task that is far beyond the capabilities of individual ants. Each single ant can detect the pheromone released by other ants when moving randomly and release its own pheromone when moving along the route, thereby increasing the number of pheromone in the path. As the number of ants increases along the way, the shortest path between food and ants will naturally form, which is the origin of the ant algorithm.

This effect can also be achieved when applied to logistics and distribution. In the initial transportation of goods, people can try multiple paths, find the path with the shortest time by timing, and mark the optimal path when they follow the same path, thereby reducing delivery time and improving delivery efficiency. In the experiments of this study, the information heuristic factor and the expected heuristic factor selection parameters will have an impact on the experimental results. In the experiment, 10 groups of experimental groups were selected, and each group selected different parameters. According to different parameters, the search situation was obtained as listed in Table 1.

According to the different values of *α* and *β*, the experiment recorded the number of effective ants and the effective time of walking the circular path. It can be seen from this that the larger the parameter value is, the smaller the number of effective ants and the longer the time-consuming. It can be seen that the more effective the number of ants to find the optimal path, the better. In addition, according to the 10 groups of experimental groups, different parameter values are the theoretical and actual distances. The comparison of theoretical distances and actual distances in the experiment is shown in Figure 9.

It can be concluded from the graph analysis that the pheromone concentration and distance heuristic information play little role in the algorithm execution process when the sum value setting is relatively small, and the searched theoretical value and the actual value are quite different. When the parameter increases gradually, the search effect gradually becomes better. The group of no. 3, *α*=2, and *β*=0.8 has the smallest gap between the theoretical shortest distance and the actual shortest distance. At this time, the influence of the pheromone concentration and the influence of the distance heuristic information are balanced, so that the algorithm can learn from the pheromone information sent by the ants before, and at the same time make reasonable use of the heuristic information.

Compared with different values of *α* and *β*, the pheromone volatility coefficient *ρ* value also affects the experimental results. The experiment selects 6 experimental groups and records the search conditions under different parameters, as listed in Table 2.

Depending on the value of *ρ*, the experiment recorded the number of effective ants and the effective duration of walking the circular path. In addition, according to the 6 groups of experimental groups, the influence of different pheromone volatilization coefficients on the information search situation was tested. The results are shown in Figure 10.

From the analysis of the experimental results, it can be seen that there are 6 groups of experimental groups according to the value of *ρ*. It can be seen from the results that the smaller the value of *ρ*, the smallest difference between the theoretical distance and the actual distance searched by the algorithm. If *ρ* is small, the virtual ant can find the best solution and can search in a wider solution space to find the best solution. In other words, we do not miss the best solution and do not blindly continue the search affecting the convergence of the algorithm.

As *ρ* gradually increases, the pheromone volatilization rate also increases. The influence of the pheromone concentration, on which the algorithm depends becomes weaker, and it is gradually controlled by the distance-inspired information, which reduces the number of possible routes and eventually converges quickly to the locally optimal solution. The opportunity to find the best practical solution is lost and the success rate of the ants reaching their destination is greatly reduced. Therefore, the value of *ρ* cannot be chosen too large. In this experiment, the experimental effect of *ρ*=0.15 is the best.

Ant colony algorithm is a new type of bionic optimization algorithm. The advantages of this algorithm are robustness, computational concurrency, positive feedback mechanism, and simple combination with other heuristic algorithms. According to different industries, the algorithm can be applied with a slight modification. In the logistics distribution industry, the shortest distance can be found, the distribution time can be effectively reduced, and the industry can follow the progress of the times.

## 5. Conclusions

Introducing intelligent management, in the current environment of massive real-time logistics information, the optimization of the distribution system path is carried out. In this study, an optimization model is established based on radio-frequency identification and ant colony algorithm, and experiments are carried out according to two methods. By comparing the results, it is concluded that the logistics distribution system supported by the intelligent management system can realize the real-time sharing of logistics location information and can also increase the route selection scheme. The shortest route can be selected from among many routes, so as to reduce transportation costs and time and provide customers with more choices. Therefore, the application of radio-frequency identification technology and ant colony algorithm in logistics will further improve the efficiency of logistics operations, further reduce the total cost of logistics, and make the development of the logistics industry more smooth.

## Figures and Tables

**Figure 1:** System frame diagram.

**Figure 2:** Flowchart of selecting the shortest path.

**Figure 3:** Working principle diagram of RFID technology.

**Figure 4:** Structure diagram of the WSID network positioning system.

**Figure 5:** Simulation diagram of ant colony action.

**Figure 6:** Localization error of the tested algorithm. (a) Target node position measurement diagram. (b) Track point fixed point error diagram.

**Figure 7:** The effect of the number of beacon nodes on localization performance.

**Figure 8:** Influence of beacon node communication distance on algorithm error.

**Figure 9:** Comparison of theoretical and actual shortest distances under different parameters.

**Figure 10:** Comparison of theoretical and actual shortest distances under different *ρ* values.

**Table 1:** Algorithm search under different parameters.

Parameter number	*α*	*β*	Effective number of ants	Operation hours (ms)
1	0.5	0.3	63	980
2	1	1	60	1185
3	2	0.8	62	867
4	2	1.2	68	1145
5	3	2	60	3245
6	4	2	58	7864
7	0.7	3	55	17650
8	2	4	54	43320
9	3	5	48	58765
10	9	9	40	57166

**Table 2:** Algorithm search under different *ρ* values.

Parameter number	*ρ*	Effective number of ants	Operation hours (ms)
1	0.15	65	830
2	0.2	60	1050
3	0.35	58	1143
4	0.5	56	954
5	0.7	50	831
6	0.85	45	837

## Data Availability

No data were used to support this study.
